# Characteristics of Lumbar Bone Density in Middle-Aged and Elderly Subjects: A Correlation Study between T-Scores Determined by the DEXA Scan and Hounsfield Units from CT

**DOI:** 10.1155/2021/5443457

**Published:** 2021-12-16

**Authors:** Dejian Zhang, Yao Wu, Shengfei Luo, Fangyong Wang, Lizhuo Li

**Affiliations:** ^1^Department of Emergency, Beijing Bo'ai Hospital, China Rehabilitation Research Center, Beijing, China; ^2^School of Rehabilitation Medicine, Capital Medical University, Beijing, China; ^3^Department of Spine and Spinal Cord Surgery, Beijing Bo'ai Hospital, China Rehabilitation Research Center, Beijing, China; ^4^Department of Rehabilitation, The Second Hospital of Tianjin Medical University, Tianjin, China; ^5^Department of Emergency, Beijing Xuanwu Hospital, Beijing, China

## Abstract

**Purpose:**

To describe the characteristics of lumbar bone density in middle-aged and elderly subjects and explore whether there is a correlation between computed tomography (CT) values and the bone mineral density (BMD) T-scores of the lumbar vertebral cancellous bone.

**Methods:**

Forty-two subjects, including 25 males and 17 females, with a mean age of 56 years, who underwent BMD measurement and lumbar multislice spiral CT scan at the China Rehabilitation Research Center from January 2019 to December 2019 were selected. Dual-energy X-ray absorptiometry (DEXA) was applied to obtain the total BMD T-scores of the lumbar L1–L4 vertebrae.

**Results:**

The CT values decreased from L1 to L4 and were 145.91 ± 8.686 HU, 143.18 ± 8.598 HU, 137.39 ± 8.276 HU, and 135.23 ± 8.219 HU, respectively. The total CT value of L1–L4 was 140.43 ± 4.199 HU. The mean total BMD T-score of L1–L4 was −0.94. The CT values of the L1–L4 vertebrae were positively correlated with the total BMD T-scores of L1–L4 (*r* = 0.349, *P* < 0.001). The CT value of the left third of the same vertebrae was the highest, and there was a strong positive correlation between the regional CT value of the lumbar spine and the entire vertebra CT values (*r* > 0.7).

**Conclusion:**

The CT values of the lumbar spine can assist the measurement of the T-scores of lumbar BMD, which could aid in early opportunistic screening for osteopenia and preventing osteoporosis and vertebral compression fractures in middle-aged and elderly subjects. This trial is registered with ChiCTR2100049571.

## 1. Introduction

Osteoporosis represents an increasing global health problem, with the highest incidence rates in postmenopausal women and elderly men [1]. Osteoporosis is a systemic bone disease characterized by osteopenia and compromised bone microstructure, resulting in increased bone fragility and susceptibility to fracture [2, 3]. It is estimated that 33% of women over 55 years old and 20% of men over 65 years old have experienced an osteoporotic fracture [4, 5]. Although we previously found that the early administration of bisphosphonate analogues is safe for improving lumbar bone mineral density (BMD), this does not appear to be effective at preventing osteoporotic fractures [6]. Therefore, early bone quality screening and thus early detection of osteopenia are important for healthy middle-aged and elderly subjects.

The clinically recognized diagnosis of osteoporosis is based on the definition of the World Health Organization (WHO) in 1994 [7]. T-scores were derived from the National Health and Nutrition Examination Survey (NHANES) III reference database for femoral neck measurements in Caucasian women aged 20–29 years [8]. The BMD T-scores measured by dual-energy X-ray absorptiometry (DEXA) in subjects with osteoporosis are −2.5 standard deviations or less relative to the average healthy young adult [9–11]. DEXA was recommended by the WHO as a gold standard for diagnosing osteoporosis. Because of its availability, relatively minimal radiation exposure, and simplicity of use, DEXA is the most commonly employed quantitative radiologic method to assess bone mass [12]. With the rapid development of computed tomography (CT) technology, it has become a promising tool for measuring BMD [13]. At present, the frequency of the application of the Hounsfield unit (HU) quantitative evaluation of local bone quality in CT scanning is increasing. The greater the bone tissue density, the higher the HU value and the lower the likelihood of a fracture [14–18].

At present, there are few studies on the regional CT values of the lumbar spine. We hypothesized that CT values of the lumbar spine are positively correlated with the BMD T-scores and that regional CT values of the lumbar spine are also positively correlated with CT values of the entire vertebra. The goals of this study were to describe the distribution characteristics of CT values and BMD T-scores of the lumbar spine in middle-aged and elderly subjects, to determine whether there was a correlation between regional CT values of the lumbar spine and those of the entire vertebra, and to describe the relationship between CT values of the lumbar spine and the BMD T-scores.

## 2. Materials and Methods

### 2.1. Participants

The study included 42 middle-aged and elderly subjects over 40 years old who received a DEXA examination in the China Rehabilitation Research Center from January 2019 to December 2019, all of whom underwent a CT scan of the lumbar L1–L4 vertebrae in our hospital during the same period (within 20 days), including 25 males and 17 females. The male-to-female ratio was 1.47. Participants ranged in age from 40 to 79 years, with a mean age of 56 years. These subjects were assigned to two age groups: 40–59 and 60–79 years. All procedures were approved by the Beijing Bo'ai Hospital Clinical Trial Organization Ethics Committee (no. 0000-0002-9499-8654).

### 2.2. Exclusion Criteria

Subjects with postoperative lumbar spine surgery, severe lumbar degenerative disease, scoliosis deformity, intravertebral tumors and infections, major diseases that may affect bone metabolism (such as congenital bone metabolism abnormalities, poliomyelitis, severe liver and kidney diseases, thyroid diseases, collagen diseases, diabetes, and bone tumors), or recent use of drugs that may affect bone metabolism were excluded from our study. All patients participated voluntarily in the study and gave written informed consent before examination.

### 2.3. Measurements

DEXA scans were performed using a Discovery Wi analyzer (Hologic, Boston, USA). The T-scores were obtained from the DEXA scan for the L1–L4 vertebrae. The instrument quality was corrected before daily measurement.

All imaging was performed using a 64-row and 128-slice multidetector CT (MDCT) scanner (Optima CT660, GE Healthcare, Chicago, USA). The CT parameters included a slice thickness of 2.0 mm, a slice interval of 1 mm, a pitch of 1.063, a tube voltage of 120 kV, and a tube current of 250 mA. All subjects were in the supine position for lumbar spine spiral scanning. The scanned images were transmitted to the workstation, and the radioactive density of the vertebral cancellous bone was measured as the HU value using a picture archiving and communication system (PACS, GE Healthcare).

There are two reasons to focus on only the measurement of cancellous bone mineral density: (1) the measurement of the cortical bone is inaccurate due to the presence of osteophytes; (2) the main pathological manifestations of osteoporosis come from the changes of the cancellous bone, that is, the thinning and fracture of cancellous bone trabeculae, the reduction or disappearance of bone trabeculae, and even microfractures. Therefore, the measurement of the lumbar cancellous bone can sensitively reflect the decline of bone mass and osteoporosis.

The cancellous bone area of the L1–4 axial pedicle plane was considered, and the nine CT measurement regions of interest were divided equally (Figure 1). Each area was set to 10.0 ± 0.2 mm^2^. In the vertical direction, the anterior third included regions 1, 2, and 3, the middle third included regions 4, 5, and 6, and the posterior third included regions 7, 8, and 9. In the horizontal direction, the left third included regions 3, 6, and 9, the center third included regions 2, 5, and 8, and the right third included regions 1, 4, and 7. The CT values of each subject were measured three times, and the mean value was taken.

### 2.4. Statistical Analyses

The level is tested according to the estimation method of sample size during quantitative data mean comparison *α* = 0.05 (one side) and inspection efficiency 1 − *β* = 0.08. According to the clinical situation and the basis of previous research and considering the skewness and accuracy of sample data, (*μ*1 − *μ*2)/SD ≌ 1.0 is determined. Finally, a total of 42 cases were determined by table lookup.

All statistical analyses were performed using Statistical Product and Service Solutions Inc. (version 25.0, Chicago, IL, USA) and Microsoft Excel (Microsoft Corporation, Redmond, WA, USA). The correlation parameters between DEXA and CT were calculated for HU values of each vertebral level from L1 to L4. The CT values are expressed as the mean ± standard deviation. The difference was defined as statistically significant in a two-sided test with *P* < 0.05. Coefficients of variance (CV) = standard deviation/mean × 100%.

Two independent samples' *t*-test was used to analyze the mean value of the L1–L4 CT and BMD T-scores in middle-aged and elderly subjects of different ages. The Spearman rank correlation test was used to detect the correlation between the lumbar spine sequence and its vertebral CT values, and a general linear model was used to test the correlation between the L1–L4 vertebral mean CT value and the corresponding vertebral total BMD T-scores. The linear correlation analysis of the CT values of each area in the L1–L4 vertebrae and the total CT values of the entire vertebrae was expressed by the Pearson correlation coefficient (0.0–0.19: very weak correlation, 0.20–0.39: weak correlation, 0.40–0.59: moderate correlation, 0.60–0.79: strong correlation, and 0.80–1.0: very strong correlation). The *r*-value range is −1 ≤ *r* ≤ 1, where *r* < 0 is a negative correlation, *r* > 0 is a positive correlation, and *r* = 0 is a nonlinear correlation.

## 3. Results

### 3.1. CT Values

The mean age of the 42 subjects was 56 years (range: 40–79 years). It was observed that the mean CT values displayed a tendency to decrease with age (*P* < 0.001) (Table 1).

In the same age range, the lumbar CT values of males and females differed. The CT value of the lumbar spine in men aged 40–59 years was significantly higher than that in women (*P* < 0.05). By contrast, there was no significant difference in the mean lumbar CT value between males and females in the elderly aged over 60 years (Table 1).

### 3.2. BMD T-Scores

According to the WHO diagnostic criteria, the T-scores of the lumbar vertebrae were classified as normal (−1.0 or greater), osteopenia (less than −1.0 and greater than −2.5), or osteoporosis (−2.5 or less) [7]. In the present study, the BMD T-score of men aged 40–59 years was in the normal range, whereas the other subjects displayed osteopenia, and the age of women with osteopenia was less than the men. The T-score of lumbar BMD in men aged 40–59 years was significantly higher than in women of that age (*P* < 0.001) (Table 1).

### 3.3. Correlation between the CT Values and T-Scores

The mean CT values for L1–L4 ranged from 135.23 HU to 145.91 HU (mean: 140.43 ± 4.20 HU), while their T-scores ranged from −1.19 to −0.72 (mean: −0.94 ± 0.09) (Table 2). For the L1–4 vertebrae, the CV for CT were 5.96, 6.01, 6.03, and 6.08, while the CV for DEXA were 14.29, 18.95, 21.35, and 27.78, respectively (Table 2). The sequence L1–4 of the lumbar spine was negatively correlated with the CT values (*r* = −0.085, *P*=0.271). With the increase of the lumbar sequence, the CT values of the cancellous bone in the vertebrae decreased gradually, whereas the BMD T-scores increased gradually.

For each lumbar spine, the correlations of the CT values and T-scores were calculated individually. For the L1–4 vertebrae, the correlation coefficients (*r*) for the CT values and T-scores were 0.538, 0.435, 0.290, and 0.220, respectively (Table 2). The total CT value of the lumbar spine was positively correlated with the total BMD T-score (*r* = 0.349, *P* < 0.001) (Table 2 and Figure 2). Therefore, it was concluded that there was a positive correlation between the CT values and T-scores of the L1–L4 vertebral cancellous bone.

### 3.4. Correlation between the Regional CT Values and Total CT Values

There were strong positive correlations between the CT values of each region in the L1–L4 vertebrae and the total CT values of the entire vertebrae, and *r* ranged from 0.739 to 0.924 (Table 3). Among the vertebrae, L1 and L2 displayed the highest correlation with region 3 (*r* = 0.924 and *r* = 0.917, respectively), L3 had the highest correlation with region 2 (*r* = 0.898), and L4 had the highest correlation with region 4 (*r* = 0.909) (Table 3).

### 3.5. Regional CT Values

There were regional differences in the CT values of each part of the vertebrae (Table 4). With the increase of the lumbar sequence, the CT values of the regional cancellous bone in the vertebrae displayed a downward trend. The CT value of the anterior third of the vertebrae was lower than that of the posterior third of the vertebrae (*P*=0.066). The CT values of different vertebrae increased gradually from right to left (*P* < 0.001). The CT value of the left third of the same vertebra was the highest.

## 4. Discussion

From the results, it was observed that the CT values of the lumbar spine correlated positively with the BMD T-scores measured by DEXA, and there was a strong positive correlation between the regional CT values of the lumbar spine and the total CT values of the same level of vertebrae, which validates our original hypothesis. Interestingly, we found that the strength of the anterior third of the lumbar vertebrae was lower than that of their posterior third in middle-aged and elderly subjects, which may at least in part explain why vertebral compression fractures often occur in the anterior column of the vertebrae.

The results showed that the CT values and T-scores of the BMD of the L1–L4 vertebrae in middle-aged and elderly subjects decreased with age, and the bone mass decreased earlier in women. The bone mass of healthy adults was reported to reach a peak when approximately 30 years old, and then the net bone mass decreased slowly and steadily with age [19]. In postmenopausal middle-aged and elderly women, because of aging and decreased sex hormone secretion, bone resorption is greater than its formation, resulting in an increased risk for osteoporosis and fracture [20]. By contrast, bone loss in men is more due to a reduction of osteogenesis, which leads to the thinning of the trabeculae [21]. The cortical bone area of males continues to increase to 60–70 years old, while the periosteum of females begins to expand from 50 years old. Elderly women display greater medullary expansion and cortical thinning due to the absorption in the cortex, exceeding that in the periosteum, which further accelerates bone loss [22].

The present study found that there was a positive correlation between the mean CT values of the L1–L4 vertebrae and the BMD T-scores calculated by DEXA in middle-aged and elderly subjects such that it can be considered that the CT values of the lumbar spine, to a certain extent, reflect the bone condition of the lumbar vertebrae. This is likely due to the fact that DEXA scan calculations include the cortex and posterior elements, whereas only the trabecular portion of the vertebra is used to determine the HU values for CT [23]. A similar result was reported in nondegenerative diseases of the lumbar spine, but the CT values of the lumbar spine can better reflect the real bone mass for patients with degenerative deformation of the lumbar spine [18, 24]. Choi et al. studied the diagnostic strength of CT values for BMD and found that, in the nondegenerative group, the CT values were strongly positively correlated with the BMD T-scores, with a correlation coefficient of *r* > 0.7, whereas in the degenerative group, there was only a weak positive correlation of *r* of approximately 0.4 [25]. A study using DEXA and quantitative CT (QCT) to measure BMD in 128 patients with low back pain found that there was a strong positive correlation between the CT values and BMD T-scores [26]. Therefore, CT can be used as an opportunistic screening tool for decreased bone density. Subjects with decreased bone density can be readily identified during routine CT scans.

The cancellous bone area of the vertebral axial pedicle plane was equally divided into nine CT measurement areas. The CT values of different regions were measured and statistically analyzed. It was found that there was a strong positive correlation between the CT values of each area and the entire vertebra, and *r* was in the range of 0.739 to 0.924. Therefore, we believe that the measurement of regional CT values in the vertebrae and BMD T-scores can preliminarily detect a decrease of bone mass. The sensitivity and specificity of the nine-zone method need to be further studied.

Further study found that there were significant differences in the CT values in different regions of the vertebrae. The CT value of the anterior third part of the vertebrae was lower than that of the posterior third, which may at least in part explain why vertebral compression fractures are more common in the anterior column of the vertebrae [27]. The most common cause of vertebral compression fracture is osteoporosis. Vertebral compression fracture secondary to osteoporosis is a cause of morbidity and even mortality in the elderly [28]. Therefore, early bone quality examination and detection of osteopenia are necessary for the prevention of osteoporosis and vertebral compression fractures.

There are several limitations in this study: (1) the number of subjects was limited, so the accuracy of the research data may have a certain degree of bias and hence the need for a large population to determine the reliability of the results. (2) In the clinic, however, surgeons may pay much attention to the preoperative bone condition of patients with lumbar degenerative diseases. It is necessary to explore the relationship between the preoperative CT values of the lumbar spine and the T-scores of the lumbar BMD in patients with lumbar degenerative diseases in a future study. (3) In this study, spiral CT was used to measure the lumbar spine CT values, but at present, QCT can more accurately measure the lumbar spine BMD [29]. Future studies can consider evaluating the correlation between the HU values measured by QCT and the T-scores determined by DEXA.

## 5. Conclusions

In brief, there was a strong positive correlation between the CT values of the lumbar spine and the BMD T-scores measured by DEXA. It is of great clinical significance to clarify the distribution characteristics of CT values and BMD T-scores of the lumbar spine in middle-aged and elderly subjects and to conduct bone quality examination at an early stage, which could aid in preventing the occurrence of osteoporosis and vertebral compression fracture. Insofar as CT is a reliable tool for measuring HU values, it can thereby be used in opportunistic screening of subjects with decreased bone density, who can then be referred for DEXA and subsequent management.

## Figures and Tables

**Figure 1:** Regional CT values of the lumbar spine were measured by the nine-zone method.

**Figure 2:** The mean CT values were positively correlated with the BMD T-scores of the L1–L4 vertebrae.

**Table 1:** Distribution of the mean CT values and BMD T-scores in the lumbar L1–L4 vertebrae.

Age (years)	Female	Male	*t*	*P*
40–59	CT value: 150.47 ± 52.75	CT value: 178.94 ± 44.90	2.761	0.007
	T-score: −1.15 ± 0.86	T-score: −0.16 ± 1.09	−4.311	＜0.001

60–79	CT value: 104.21 ± 36.26	CT value: 97.39 ± 19.24	−0.996	0.324
	T-score: −1.56 ± 1.22	T-score: −1.15 ± 1.26	−1.405	0.164

**Table 2:** Correlation between the CT values and BMD T-scores in different lumbar sequences.

Lumbar sequences	CT		DEXA		*r*	*P*
	CT values (HU)	CV (%)	BMD T-scores	CV (%)		
L1	145.91 ± 8.69	5.96	−1.19 ± 0.17	14.29	0.538	＜0.001
L2	143.18 ± 8.60	6.01	−0.95 ± 0.18	18.95	0.435	0.004
L3	137.39 ± 8.28	6.03	−0.89 ± 0.19	21.35	0.290	0.062
L4	135.23 ± 8.22	6.08	−0.72 ± 0.20	27.78	0.220	0.161
Average	140.43 ± 4.20	2.99	−0.94 ± 0.09	9.57	0.349	＜0.001

CV: coefficients of variance.

**Table 3:** Correlation between the regional CT values and the total CT values in different lumbar sequences.

Different regions	Correlation coefficient in different lumbar sequences (*r*)			
	L1	L2	L3	L4
Region 1	0.868	0.827	0.857	0.757
Region 2	0.886	0.895	0.898	0.844
Region 3	0.924	0.917	0.835	0.831
Region 4	0.866	0.806	0.818	0.909
Region 5	0.875	0.862	0.863	0.854
Region 6	0.844	0.828	0.778	0.739
Region 7	0.895	0.862	0.860	0.885
Region 8	0.918	0.914	0.879	0.895
Region 9	0.862	0.856	0.803	0.874

**Table 4:** Regional CT values in different lumbar sequences.

Lumbar sequences	Vertical (HU)			Horizontal (HU)		
	Anterior 1/3	Middle 1/3	Posterior 1/3	Left 1/3	Center 1/3	Right 1/3
L1	136.38 ± 4.42	148.25 ± 4.89	147.4 ± 5.22	154.20 ± 5.30	145.19 ± 4.81	132.64 ± 4.27
L2	136.38 ± 4.61	143.21 ± 5.02	139.61 ± 4.98	146.66 ± 5.14	142.09 ± 4.88	130.44 ± 4.48
L3	131.80 ± 4.56	134.66 ± 4.76	134.15 ± 4.99	138.44 ± 4.90	137.56 ± 4.78	124.60 ± 4.54
L4	130.90 ± 4.92	137.28 ± 4.90	139.53 ± 5.10	139.70 ± 5.13	138.30 ± 4.92	129.71 ± 4.85
Average	133.86 ± 2.31	140.85 ± 2.45	140.17 ± 2.54	144.75 ± 2.57	140.79 ± 2.42	129.35 ± 2.27

## Data Availability

The datasets used during the current study are available from the corresponding author upon reasonable request.
